# Shoe Bending Stiffness Influence on Lower Extremity Energetics in Consecutive Jump Take-Off

**DOI:** 10.1155/2022/5165781

**Published:** 2022-05-29

**Authors:** Sheng-Wei Jia, Fan Yang, Yi Wang, Tongtong Guo, Wing-Kai Lam

**Affiliations:** ^1^Li Ning Sports Science Research Center, Li Ning (China) Sports Goods Company Limited, Beijing 101111, China; ^2^Department of Physical Education and Research, China University of Mining and Technology-Beijing, 100083 Beijing, China; ^3^Department of Physical Education, Renmin University of China, 100872 Beijing, China; ^4^Sports Information and External Affairs Centre, Hong Kong Sports Institute, Sha Tin, Hong Kong

## Abstract

**Objective:**

This study examined the influence of shoe bending stiffness on lower extremity energetics in the take-off phase of consecutive jump.

**Methods:**

Fifteen basketball and volleyball players wearing control shoes and stiff shoes performed consecutive jumps. Joint angle, angular velocity, moments, power, jump height, take-off velocity, take-off time, and peak vertical ground reaction force data were simultaneously captured by motion capture system and force platform. Paired *t*-tests were performed on data for the two shoe conditions that fit the normal distribution assumptions, otherwise Wilcoxon signed-rank tests.

**Results:**

There are significant differences (*P* < 0.05) in take-off velocity and take-off time between stiff and control shoe conditions; the stiff shoes had faster take-off velocity and shorter take-off time than control shoes. There was no significant difference between two conditions in jump height (*P* = 0.512) and peak vertical ground reaction force (*P* = 0.589). The stiff shoes had significantly lower MTP dorsiflexion angle and greater joint work than the control shoes (*P* < 0.05). The MTP range of motion and maximum angular velocity in stiff shoe condition were significantly lower than those in control shoe condition (*P* < 0.01). However, there are no significant differences between two conditions in kinetics and kinematics of the ankle, knee, and hip joint.

**Conclusions:**

The findings suggest that wearing stiff shoes can reduce the effect of participation of the MTP joint at work and optimize the energy structure of lower-limb movement during consecutive jumps.

## 1. Introduction

In basketball and volleyball, jumping is important and frequently executed which can be the determining factor for the outcome of a game [1, 2]. The repetitive and rapid jumps were required for rebound and block movements in basketball [3]. The previous study suggests that compared to a single jump, the consecutive jump is closer to realistic competition and provides more meaningful information to sports trainers [4]. Therefore, improving the consecutive jump ability appears necessary for basketball and volleyball players.

Previous studies have focused on improving the ability to jump through training methods [5, 6]. Markovic and colleagues [7] suggested that plyometric training could promote the use of the elastic energy and neural response benefits during the stretch-shortening cycle. Struzik and Zawadzki found that the take-off velocity is related to the stiffness of the legs, and the legs with higher stiffness have better take-off velocity performance [8]. Studies have also found a positive correlation between the take-off velocity and the MTP joint stiffness in the consecutive jump [9]. Faster take-off velocities shorten the time to reach the highest point, which makes the athlete more competitive in the race [3]. However, some studies have found that changes in footwear can affect the biomechanical characteristics [10] and jump performance. Brizuela and colleagues [11] found that increased ankle support in high-top shoes reduces ankle valgus range but increases shock to the body and reduces jumping ability.

The bending stiffness of the shoe midsole has been suggested to be a direction to influence jump performance [12, 13]. One study found that MTP joint has no energy generation but absorbs large amounts of energy during take-off [14]. When increasing the midsole stiffness, a stiffer midsole would minimize the energy loss at the MTP joints, it significantly optimized the performance of the lower extremities [12]. A similar conclusion was found in another study, which found that the jump height of shoes with medial and lateral plates was higher than that of only medial plate or without it [13].

Moreover, a previous study suggested that increasing longitudinal bending stiffness of the midsole can reduce the muscle activity required to perform negative work, resulting in overall improved running economy [15]. Tinoco et al. [16] indicated that the stiffer midsole can effectively compensate for the decline in jump performance caused by fatigue.

However, the effect of bending stiffness was inconsistent between studies with different plates and types of jump. The research suggested that increasing the stiffness from flexible to the stiff conditions would not induce a beneficial effect on jump height, suggesting that the height of a single jump is not sensitive to shoes with minor differences in the bending stiffness [17]. Furthermore, extremely high bending stiffness may increase the risk of injury. High bending stiffness cycling shoes (SH-M220, Shimano, Osaka, Japan) have been shown to generate more discomfort in nonprofessional cyclists and aggravate disease in the metatarsal area, as indicated by the higher peak plantar pressure [18]. Consequently, the limited MTP flexion may be the plausible reason to increase the plantar pressure, which leads to aggravate metatarsalgia or ischaemia syndromes [18]; it also suggested that extremely high bending stiffness was not suitable for nonprofessional players.

Most studies on shoe bending stiffness are limited to single jumps and the effect on the lower extremities during the consecutive jumps. Rebounding and blocking in basketball often require repetitive and quick jumps [3]. The consecutive jump is considered to be closer to the realistic competition and can provide more meaningful information to the sports trainers than the single jumps [4]. Consecutive jumps can represent the explosive power of the lower body [19]. Furthermore, there are some biomechanical differences between single CMJ and consecutive jump. When comparing the two movements, consecutive jumps showed higher MTP and ankle extension angular velocity. The ankle, knee extension power, and knee extension moment were greater in consecutive jumps [2]. Therefore, the effect of midsole bending stiffness on consecutive jump and lower-limb biomechanics needs to be further explored.

Athletes and footwear manufacturers have long been interested in the effects of shoes on jump performance [20]. Previous studies on the effect of shoe bending stiffness on the lower limb in consecutive jumps are limited. Moreover, in consecutive jumps, the effect of shoe midsole stiffness on lower extremity chain biomechanics, jump height, or take-off velocity remains unclear. The objective of the study is to explore the influence of different bending stiffness of the midsole on jump performance and biomechanical characteristics on lower extremities in consecutive jumps. It is expected that wearing higher bending stiffness shoes limits the range of motion (RoM) and angular velocity in the MTP joint and at the same time increases the RoM in the ankle and knee joints and joint energetics and jump height performance.

## 2. Materials and Methods

### 2.1. Shoe Conditions

Two conditions of shoes (stiff and control) were used in this study. The control shoe was the commercially available model for professional basketball players (ABAS011, Li-Ning, Beijing, China), which had a removable midsole (i.e., combined the insole and midsole) (Figures 1(a) and 1(b)). The stiff shoe condition was identical to the control shoe, except that there is a full-length carbon plate under the removable midsole, so that it lay between the midsole and the outsole (Figure 1(b)). This is thought to minimize discomfort and not to damage the shoe construction, which could be the contributing factors to jump performances and movement mechanics. The forefoot area of the shoe was fixed by the toe cap fixture, and the forefoot of the shoe was flexed from 0 degree (horizontal) to 45 degrees at 70% of the shoe length in alignment with the bending axis of the mechanical flexion tester (F911-85, ASTM, West Conshohocken, USA) (Figure 2). A total of 65 flexion trials were performed for each shoe condition, and the average value was taken from the last five trials to represent the bending stiffness of the control shoe and the stiff shoe.

### 2.2. Participants

A priori power analysis was calculated by G∗power (version 3.1.9.7; Heinrich Heine University, Germany) with a power of 0.8, indicating that a minimum number of 15 participants were required. Therefore, we recruited 15 male collegiate basketball or volleyball players (age = 21.2 ± 1.3 yrs; height = 176.7 ± 3.5 cm; body mass = 73.4 ± 5.6 kg; shoe size = 9 US) with 5.5 ± 1.2 yrs of experience in basketball or volleyball for this research. The dominant leg of all participants is the right leg, the way to distinguish the dominant leg is to instruct the participant to kick the ball at 4 m ahead, and if the participant kicks the ball with the right foot, then the right leg is defined as the dominant leg [21]. All participants have no lower extremity injuries, at least in the last six months. The experimental procedure was approved by the Li Ning Institutional Ethics Committee, and all participants signed informed consent.

### 2.3. Procedure

On arrival, the participants were briefed with the project information and signed an informed consent form. We performed anthropometric measurements including height, weight, standing touch height, foot length, and foot width. 22 reflective markers with a radius of 7 mm are distributed on the hip (four markers), right thigh (four-marker cluster), right knee joint (two markers), right shank (four-marker cluster), right ankle joint (two markers), and right foot (six markers) [2] (refer to Figure 3 for the specific location of markers).

Participants warm up with five-minute treadmill run at a personal comfortable pace, followed by self-administrated stretches and some jumps [22].

The participants were asked to put on standard socks and test shoes, which were randomly selected. At the start of consecutive jumping task, participants were asked to place right leg stand on the force platform and the left leg on the surrounding floor. Participants performed five consecutive jumps in a row without an obvious pause after each landing and require to immediately start the next jump [23]. They were required to keep the right foot on the same force platform during five consecutive jumps, and the left foot was not in contact with the force plate. A period of 120 s rest after each trial completes a shoe condition after successfully collecting valid data for 3 times consecutive jumps.

All athletes performed consecutive jump sessions. Countermovement jump is commonly used to assess lower body explosiveness and jumping performance in sports. It is also a key movement in biomechanical studies related to basketball shoes [13, 24–26]. All experimental data were simultaneously captured by an 8-camera Vicon system (200 Hz, Oxford Metrics Ltd, Oxford, UK) and a 3D force plate (1000 Hz, AMTI, Watertown, USA). The collected data included lower extremity joints' angle, angular velocity, RoM, moment, power, work, take-off velocity, jump height, take-off time, and GRF data.

### 2.4. Data Processing

The force data and marker trajectory data of the participants in the experiment were collected and recorded synchronously by operating Vicon Nexus software (Oxford Metrics Ltd, Oxford, UK). After the marker naming process, export the file to Visual 3D software (C-Motion Inc., Germantown, USA) to calculate and output all the required indicators. The kinematic data were processed with a 12 Hz cut-off Butterworth fourth-order low-pass filter [27]. The take-off period of kinetics and kinematics is defined as the time from the lowest midpoint of the line connecting the two posterior superior iliac spines (CoM) to the moment when the toes lift off the ground (the vertical GRF first drops to 10 N) [23, 28] (Figure 4). The take-off period of the jump performance is the period from the lowest to the highest point of CoM (Figure 4). The jump height calculation method is the difference between the highest point of CoM after take-off and CoM when standing still [29, 30]. The take-off velocity is calculated with reference to the upward speed of CoM after the feet leave the ground [31]. Joint angle, angular velocity, RoM, moment, power, and work are calculated by Visual 3D software. The moment, power, and work are calculated using the inverse dynamic model method [12, 13, 32] and standardized by body height (BH) and body weight (BW). The GRF data were standardized by body weight (BW). The zero degree of joint was defined in the static standing position. Hip flexion, knee extension, ankle dorsiflexion, and MTP dorsiflexion were uniformly defined as positive values.

### 2.5. Data Analysis

Considering that the first jump of the consecutive jump is a single jump in nature and different from the rest of the trials, only the second to fourth jump trials were extracted for subsequent analysis (Figure 4). Data normality was firstly examined with the Shapiro-Wilk test. Paired *t*-tests were performed on jumping performance, kinematics, and kinetic data for the two shoe conditions that fit the normal distribution assumptions, otherwise Wilcoxon signed-rank tests. Data were analyzed with SPSS software (SPSS 22.0, SPSS Inc., Chicago, USA). The significance level was set at *α* = 0.05. The effect size result was interpreted as follows: the range of small effect is 0.2 to 0.5, medium effect is 0.5 to 0.8, and large effect is more than 0.8 [33].

## 3. Results

### 3.1. Shoe Bending Stiffness

Through measurement, the bending stiffness of the control shoe is 0.297 Nm/°, and the bending stiffness of the forefoot of the hard-soled shoe is 0.366 Nm/° (Table 1).

### 3.2. Jump Performance and GRF Variables

The take-off velocity was significantly faster in the stiff shoe condition (*P* < 0.05, *d* = −2.85, medium effect); the take-off time of the stiff shoe condition is significantly shortened (*P* < 0.05, *r* = 2.19, small effect) (Table 2).

### 3.3. Kinematics and Kinetics of the MTP, Ankle, Knee, and Hip Joints

The stiff shoe condition had significantly lower MTP joint dorsiflexion angle (*P* < 0.05, *d* = 2.41, medium effect), RoM (*P* < 0.01, *d* = 3.53, large effect), and maximum angular velocity (*P* < 0.01, *d* = 6.94, large effect), and the work was greater than control shoe (*P* < 0.05, *d* = 2.23, large effect) (Table 3).

No significant differences between two conditions were found in hip, knee, and ankle joints (Table 3).

## 4. Discussion

This study investigated the biomechanical effects of consecutive jumps with two different conditions of forefoot bending stiffness as a reference for jumping-related sports. The experimental results supported part of our hypothesis that the stiff shoe condition restricted the RoM and the joint angular velocity of the MTP joint during the take-off period. But there is no significance in kinematics and kinetics of ankle, knee, and hip joint, as well as jump height.

The jump height results did not support our hypothesis, which is also different from Stefanyshyn and Nigg's findings [14]. The authors suggested that the stiffer shoes reduce the energy absorbed from the MTP joint, and the rest of energy would improve about 3.5 cm height (70 kg mass body). Some other studies also found no significant differences between stiff and control conditions in lay-up movement [22] and running vertical jumps [17]. One possible reason is that the actual difference in stiffness between the two shoes is too small to generate the significant improvement showed in Stefanyshyn and Nigg's study (energy improvement = mass × height × gravity = 70 × 3.5/100 × 9.81); the experiment of Stefanyshyn and Nigg's [12] research increased the forefoot stiffness from 0.04 Nm/° to 0.25 Nm/°; our conditions only compared the difference between 0.297 Nm/° and 0.366 Nm/°, so it is not difficult to understand: there are significant differences in MTP joint work, but insufficient changes at the MTP joint to significantly alter athletic performance. However, according to our results, the stiff shoes significantly improved the take-off velocity and shortened the take-off time, which are considered to be positive performance benefit in sports [3]. Faster take-off velocity can help an offensive player disrupt the defender's timing, create a foul, and then take a shot [34]. This is similar to previous studies, who also found that higher forefoot bending stiffness improved sprint and cut performances [13, 17].

As hypothesized, several differences in MTP kinematics were found. These changes are in line with the previous research [12, 14]. Increasing MTP joint stiffness reduced MTP joint maximum dorsiflexion angle and RoM, limited the angular velocity of MTP joint dorsiflexion, and minimized dissipated energy, which is related to improved jump velocity. These confirm our previous first hypothesis. Joints with greater angular velocity and loading represent greater range of motion and muscle-ligament strain in rapid push-off, which may suggest better take-off performance [9]. It should be noted that it would also be considered potentially modifiable risk factors for lower extremity injuries [35, 36]. At the instant before toe-off the ground, the MTP plantarflexion angular velocity in the stiff shoe condition is higher than that in the control condition. Although there is no statistical difference, it can be explained to a certain extent that a shoe with high stiffness might restore the forefoot to its original position faster [37].

From the test results, there is no significant difference in the kinematics and kinetics of the hip, knee, and ankle joints, which does not agree with some literatures. The results of Zhu and colleagues [22] showed that a stiff midsole significantly improved ankle RoM, maximum power, energy absorbed, and energy produced. Another study also found that stiff shoes can regulate the biomechanical properties of the ankle joint [38]. They believe that the stiff shoe changes the force application point to the position where the toe region is in contact with the ground, resulting in the occurrence of a complementary change of the lower extremity joint kinematic chain. No such obvious changes determined in this paper may be due to the small change in the stiffness of the midsole [17], and it is also possible that compared with a single jump (MTP angle is zero at the beginning), after the buffer stage of the last landing, the forefoot has been bent at the beginning of the take-off stage, resulting in a small change in GRF application point.

Through this experiment and combined with previous studies on vertical jumps [12, 22], the effect of shoe bending stiffness on the upward jump is concentrated on the MTP joints, and the influence on the hip and knee joints is relatively small.

There are some limitations in this study. There are only two conditions in this study. If there are more stiffness carbon plates with larger absolute differences between shoe conditions, the systematic changes can be established for a deeper interpretation. Moreover, only the collegiate basketball and volleyball team players were recruited; the professional athletes would be used to evaluate the shoe bending effect as indicated by consistent jump movements between trials in professional athletes.

## 5. Conclusions

During the five consecutive jumps, the longitudinal midsole stiffness would significantly improve the take-off speed and shorter time to reach the highest point but did not result in the absolute difference in jump height and lower-limb joint kinematics. These results suggest that wearing stiff shoe can reduce the effect of MTP joint participation in work and optimize the energy structure of lower-limb movement during consecutive jumps.

## Figures and Tables

**Figure 1:** Schematic diagram of shoe conditions: (a) control shoe; (b) stiff shoe.

**Figure 2:** Shoe bending stiffness tester.

**Figure 3:** Reflective markers scheme: (a) right view; (b) left view.

**Figure 4:** Data analysis area in consecutive jump.

**Table 1:** Shoe bending stiffness.

Variables	Control shoe	Stiff shoe
Shoe bending stiffness (Nm/°)	0.297	0.366

**Table 2:** Jump performance and GRF variables (mean ± SD).

Variables	Control shoe	Stiff shoe	*T*/*Z*	*P*	Effect size
Take-off velocity (m/s)	2.68 ± 0.15	2.74 ± 0.17	-2.85	*0.013*	0.74
Jump height (BH)	0.28 ± 0.02	0.28 ± 0.02	0.67	0.512	0.17
Peak GRF (BW)	1.30 ± 0.35	1.32 ± 0.28	0.54^Z^	0.589	0.00^a^
Take-off time (s)	0.28 ± 0.02	0.27 ± 0.02	2.19^Z^	*0.028*	0.36^a^

^a^Wilcoxon signed-rank test was performed using *r*, otherwise paired *t*-test was performed using Cohen's *d*. *Z* represents the *Z*-value, otherwise it is the *T*-value. Italic numbers indicate significant difference between two conditions.

**Table 3:** Kinematics and kinetics of the MTP, ankle, knee, and hip joints during the take-off phase (mean ± SD).

Variables	Control shoe	Stiff shoe	*T*/*Z*	*P*	Effect size
MTP					
Max. angle (°)	36.96 ± 2.88	35.14 ± 2.29	2.41	*0.030*	0.62
Min. angle (°)	28.46 ± 3.34	28.62 ± 2.30	-0.25	0.808	0.06
RoM (°)	8.50 ± 1.84	6.52 ± 2.19	3.53	*0.003*	0.91
Max. angular velocity (°/s)	164.97 ± 44.72	129.36 ± 33.96	6.94	*0.000*	1.79
Min. angular velocity (°/s)	−252.29 ± 75.44	−272.50 ± 74.00	2.02	0.064	0.52
Max. moment (Nm/BW·BH)	0 ± 0.02	0 ± 0.02	1.54^Z^	0.125	0.56^a^
Min. moment (Nm/BW·BH)	−0.17 ± 0.09	−0.17 ± 0.05	0.10	0.923	0.03
Max. power (W/BW·BH)	0.31 ± 0.13	0.27 ± 0.13	1.40	0.183	0.36
Min. power (W/BW·BH)	−0.34 ± 0.19	−0.21 ± 0.15	1.51^Z^	0.132	0.55^a^
Work (J/BW·BH)	−0.01 ± 0.01	0 ± 0.01	2.23^Z^	*0.026*	0.97^a^
Ankle					
Max. angle (°)	28.09 ± 5.71	28.15 ± 5.94	-0.11	0.911	0.03
Min. angle (°)	−39.08 ± 6.46	−39.58 ± 6.82	0.84	0.414	0.22
RoM (°)	67.17 ± 6.56	67.73 ± 6.83	-0.86	0.402	0.22
Max. angular velocity (°/s)	−775.61 ± 108.52	−775.85 ± 117.93	0.02	0.982	0.01
Max. moment (Nm/BW·BH)	0.02 ± 0.02	0.01 ± 0.02	0.92	0.371	0.24
Min. moment (Nm/BW·BH)	−0.90 ± 0.22	−0.89 ± 0.17	-0.21	0.834	0.06
Max. power (W/BW·BH)	6.11 ± 2.16	6.03 ± 1.50	0.20	0.845	0.05
Min. power (W/BW·BH)	−0.34 ± 0.34	−0.35 ± 0.28	0.51^Z^	0.609	0.03^a^
Work (J/BW·BH)	0.46 ± 0.14	0.48 ± 0.10	-0.39	0.701	0.10
Knee					
Max. angle (°)	−16.40 ± 22.03	−18.07 ± 11.62	0.34^Z^	0.733	0.26^a^
Min. angle (°)	−100.97 ± 19.16	−102.17 ± 20.88	0.72	0.486	0.19
RoM (°)	78.30 ± 19.75	83.57 ± 16.89	-1.21	0.247	0.31
Max. angular velocity (°/s)	879.54 ± 111.67	868.46 ± 112.65	0.84	0.414	0.22
Max. moment (Nm/BW·BH)	1.34 ± 0.33	1.34 ± 0.34	0.04	0.973	0.01
Min. moment (Nm/BW·BH)	−0.23 ± 0.12	−0.23 ± 0.11	0.18	0.862	0.05
Max. power (W/BW·BH)	8.79 ± 1.65	8.59 ± 1.44	0.76	0.461	0.20
Min. power (W/BW·BH)	−3.49 ± 2.02	−3.64 ± 1.79	0.29	0.777	0.07
Work (J/BW·BH)	0.79 ± 0.212	0.83 ± 0.23	1.02^Z^	0.306	0.26^a^
Hip					
Max. angle (°)	78.85 ± 22.40	79.84 ± 22.43	-0.52	0.609	0.14
Min. angle (°)	18.16 ± 19.62	17.16 ± 14.28	1.25^Z^	0.211	0.21^a^
RoM (°)	55.55 ± 16.33	60.15 ± 15.89	-1.75	0.101	0.45
Max. angular velocity (°/s)	−446.32 ± 83.70	−454.65 ± 76.96	0.57^Z^	0.580	0.15^a^
Max. moment (Nm/BW·BH)	0.26 ± 0.13	0.30 ± 0.16	-1.25	0.234	0.32
Min. moment (Nm/BW·BH)	−1.20 ± 0.23	−1.29 ± 0.24	1.42	0.178	0.37
Max. power (W/BW·BH)	3.50 ± 0.83	3.76 ± 1.10	-1.97	0.069	0.51
Min. power (W/BW·BH)	−2.50 ± 1.36	−3.03 ± 1.47	1.79	0.095	0.46
Work (J/BW·BH)	0.37 ± 0.16	0.39 ± 0.23	-1.00	0.333	0.26

^a^Wilcoxon signed-rank test was performed using *r*, otherwise paired *t*-test was performed using Cohen's *d*. *Z* represents the *Z*-value, otherwise it is the *T*-value. Italic numbers indicate significant difference between two conditions.

## Data Availability

The data used to support the findings of this study are available from the corresponding author upon request.
